The article "High expression level and nuclear localization of Sam68 are associated with progression and poor prognosis in colorectal cancer" was retracted in 2021. Reasons: duplicated images; unreliable results or conclusions; concerns about the data; concerns about the images.

# High expression level and nuclear localization of Sam68 are associated with progression and poor prognosis in colorectal cancer

**DOI:** 10.1186/1471-230X-13-126

**Published:** 2013-08-09

**Authors:** Wen-Ting Liao, Jun-Ling Liu, Zheng-Gen Wang, Yan-Mei Cui, Ling Shi, Ting-Ting Li, Xiao-Hui Zhao, Xiu-Ting Chen, Yan-Qing Ding, Li-Bing Song

**Affiliations:** 1 Department of Pathology, Nanfang Hospital, Southern Medical University, Guangzhou, Guangdong 510515, China; 2 State Key Laboratory of Oncology in Southern China, Department of Experimental Research, Sun Yat-sen University Cancer Center, Guangzhou, Guangdong 510060, P.R. China; 3 Department of Pathology, School of Basic Medical Sciences, Southern Medical University, Guangzhou 510515, China; 4 State Key Laboratory of Oncology in South China, Department of Medical Oncology, Sun Yat-sen University Cancer Center, Guangzhou, Guangdong 510060, China; 5 Department of Gastroenterology, the Second Affiliated Hospital, University of South China, HengYang, Hunan 421000, China

**Keywords:** Sam68, Biomarker, Prognosis, Colorectal cancer

## Abstract

**Background:**

Src-associated in mitosis (Sam68; 68 kDa) has been implicated in the oncogenesis and progression of several human cancers. The aim of this study was to investigate the clinicopathologic significance of Sam68 expression and its subcellular localization in colorectal cancer (CRC).

**Methods:**

Sam68 expression was examined in CRC cell lines, nine matched CRC tissues and adjacent noncancerous tissues using reverse transcription (RT)-PCR, quantitative RT-PCR and Western blotting. Sam68 protein expression and localization were determined in 224 paraffin-embedded archived CRC samples using immunohistochemistry. Statistical analyses were applied to evaluate the clinicopathologic significance.

**Results:**

Sam68 was upregulated in CRC cell lines and CRC, as compared with normal tissues; high Sam68 expression was detected in 120/224 (53.6%) of the CRC tissues. High Sam68 expression correlated significantly with poor differentiation (*P* = 0.033), advanced T stage (*P* < 0.001), N stage (*P* = 0.023) and distant metastasis (*P* = 0.033). Sam68 nuclear localization correlated significantly with poor differentiation (*P* = 0.002) and T stage (*P* =0.021). Patients with high Sam68 expression or Sam68 nuclear localization had poorer overall survival than patients with low Sam68 expression or Sam68 cytoplasmic localization. Patients with high Sam68 expression had a higher risk of recurrence than those with low Sam68 expression.

**Conclusions:**

Overexpression of Sam68 correlated highly with cancer progression and poor differentiation in CRC. High Sam68 expression and Sam68 nuclear localization were associated with poorer overall survival.

The article "High expression level and nuclear localization of Sam68 are associated with progression and poor prognosis in colorectal cancer" was retracted in 2021. Reasons: duplicated images; unreliable results or conclusions; concerns about the data; concerns about the images.

## Background

Colorectal cancer (CRC) is one of the most prevalent malignancies worldwide. Although advances have been made in diagnostic and therapeutic techniques, the prognosis of CRC patients with distant metastases still remains poor [1]. Thus, characterization of the molecular mechanism that involves in progression and metastasis of CRC could help to identify specific biomarkers which may facilitate efficient therapeutic stratification, prediction and disease prevention.

Src-associated in mitosis, 68 kDa (Sam68) belongs to the signal transduction and activation of RNA (STAR) family of K homology (KH) domain-containing RNA binding proteins [2] and is originally identified as a substrate for Src kinase phosphorylation during mitosis [3,4]. Sam68 is ubiquitously expressed and plays important roles in signaling transduction, gene transcription, and alternative splicing [2,5]. Sam68 has been suggested to act as an adaptor in signal transduction by binding to SH3- and SH2-containing proteins, through its proline-rich regions [6]. Additionally, Sam68 can interact with signaling proteins, such as Src, Grb2, Grap, SHP-1, PLCγ1/Fyn, BRK and PI3K, and has been implicated in T-cell receptor and insulin receptor signaling, as well as Ras and PI3K kinase pathways [7-11]. Moreover, Sam68 is usually a nuclear protein and plays a major role in the regulation of RNA metabolism, including mRNA transcription, alternative splicing and nuclear export [12-17]. The alternative splicing of multiple genes regulated by Sam68, including those involved in oncogenesis, such as CD44, Bcl-xl, Sgce, SMN2, SF2/ASF and Cyclin D1 [6,14-19].

The above mentioned biological functions of Sam68 closely linked this protein to oncogenic properties. First, Sam68 is involved in promotion of cell cycle progression, cell proliferation, transformation, tumorigenesis and metastasis in different cellular context [20-25]. Second, a series of published articles in the recent decade have demonstrated that Sam68 participates in transcriptional and post-transcriptional regulation of gene expressions that are relevant to human cancer [14,15,17,18,20,26]. However, deregulation of Sam68 in human cancer tissues has only been observed in limited cancer types, including prostate cancer, renal cell carcinoma, breast and cervical cancer [23,24,26-28]. Whether the deregulation of Sam68 is a prevalent event in human cancer needs further investigation. To explore the deregulation of Sam68 in human colorectal cancer, we investigated the expression patterns of Sam68 in human CRC tissues, and the correlation between Sam68 expression levels and the clinicopathologic features of CRC. Our current study indicates that the expression and localization of Sam68 may act as independent biomarkers of prognosis in CRC, suggesting that Sam68 has potential as a novel therapeutic target for the treatment of CRC.

The article "High expression level and nuclear localization of Sam68 are associated with progression and poor prognosis in colorectal cancer" was retracted in 2021. Reasons: duplicated images; unreliable results or conclusions; concerns about the data; concerns about the images.

## Methods

### Cell lines

Colorectal cancer cell lines including LS174t, Colo205, SW480, HT29, HCT116 and SW620 cells were cultured in RPMI 1640 (Invitrogen, Carlsbad, CA, USA) supplemented with 10% fetal bovine serum, 100 μg/μL streptomycin and 100 μg/μL penicillin in a humidified incubator containing 5% CO_2_ at 37°C.

### Patients and tissue specimens

For the use of clinical materials for research purposes, prior patients' consents and approval were obtained from the Sun Yat-sen University and Cancer Center Institutional Board. All samples were collected and analyzed with prior written informed consents from the patients. A total of 224 paraffin-embedded colorectal cancer samples, which were histopathologically and clinically diagnosed at the Sun Yat-sen University Cancer Center between the year 2000 to 2003, were examined. All of the patients had received chemotherapy after surgery. Prior patient consent and approval were obtained from the Institutional Research Ethics Committee.

The clinicopathological features of the patients are summarized in Additional file 1: Table S1. The final study population included 97 female and 127 male patients (age range, 23–82 years). Follow-up was recorded from the date of surgery until death. Patients who died of cancer (or other causes) were classified as dead. The median follow-up time for all patients was 58.47 months. 43 corresponding metastatic lymph nodes were also obtained from the above mentioned patients. Four pairs of CRC biopsies and the matched adjacent non-cancerous colon tissues were obtained from each patient during surgery, and immediately frozen and maintained in liquid nitrogen until further use.

### RNA extraction, reverse transcription-polymerase chain reaction and quantitative Real-time polymerase chain reaction

Total RNA was extracted from the cultured cells and surgical tissues using TRIzol reagent (Invitrogen) according to the manufacturer's instructions. Reverse transcription polymerase chain reaction (RT-PCR) and quantitative real-time polymerase chain reaction (Q-PCR) analysis of Sam68 expression were performed as previously described [29], using previously published primers and probes [28]. Sam68 expression was analyzed using the 2^-∆∆Ct^ method as described by Livak et al. [30] and normalized to the geometric mean expression level of the housekeeping gene glyceraldehyde-3-phosphate dehydrogenase (GAPDH). The relative change in Sam68 expression was calculated by pair-wise comparison of the normalized Sam68 expression level in the tumor samples with the adjacent non-cancerous tissue samples from the same patient.

The article "High expression level and nuclear localization of Sam68 are associated with progression and poor prognosis in colorectal cancer" was retracted in 2021. Reasons: duplicated images; unreliable results or conclusions; concerns about the data; concerns about the images.

### Western blotting

Tissue and cell lysates were prepared using SDS lysis buffer and the protein concentration was determined using the Bradford assay (Bio-Rad Laboratories, Hercules, CA, USA). Equal amounts of protein were separated by electrophoresis on a 10.5% sodium dodecyl sulfate polyacrylamide gel and electrotransferred from the gel to a nitrocellulose membrane. After blocking with 5% milk solution in Tris-buffered saline with Tween (TBST) for 1 hour, the membrane was incubated with primary antibody against rabbit antibody Sam68 (sc-333, dilution, 1:500; Santa Cruz Biotechnology, CA, USA) and rabbit anti-α-Tubulin (1:1000, Sigma, Saint Louis, MI, USA) primary antibodies. After washing with TBS-T, the membrane was incubated with secondary antibody against rabbit immunoglobulin G or mouse immunoglobulin G; then, it was examined with the enhanced chemiluminescence detection system (Amersham Biosciences Europe, Freiberg, Germany) according to the manufacturer’s instructions.

### Immunohistochemistry

Paraffin sections were deparaffinized with xylene and rehydrated, then submerged into EDTA antigenic retrieval buffer and microwaved for antigenic retrieval. The sections were then treated with 3% hydrogen peroxide in methanol to quench the endogenous peroxidase activity, followed by incubation with 1% BSA to block the non-specific binding. The sections were incubated with rabbit anti-Sam68 (sc-333, dilution, 1:500; Santa Cruz Biotechnology, CA, USA) overnight at 4°C. As negative controls, rabbit anti-Sam68 antibody was replaced with normal goat serum, or the rabbit anti-Sam68 antibody was blocked by co-incubation with a recombinant Sam68 polypeptide at 4°C overnight prior to the immunohistochemical staining. The staining intensity was scored on a scale of 0 to 3 as 0 (no staining), 1 (weak staining ~ light yellow), 2 (moderate staining ~ yellowish brown) or 3 (strong staining ~ brown). Tumors with a staining intensity ≥ 2 in which at least 50% of the malignant cells were Sam68-positive were classified as high expression; tumors with a staining intensity < 2 or in which less than 50% of the malignant cell were Sam68-positive were classified as low expression.

### Statistical analysis

All statistical analyses were carried out using SPSS 10.0 (Chicago, IL, USA). The significance of the differences between the normal and tumor tissue Q-PCR results were assessed using the Student’s two-tailed *t*-test. The association between Sam68 expression and clinicopathological variables were assessed using the Mann–Whitney U test. Survival curves were plotted using the Kaplan-Meier method. The Cox proportional hazards regression model was used for univariate and multivariate analysis. Two-tailed *P* values < 0.05 were considered significant.

The article "High expression level and nuclear localization of Sam68 are associated with progression and poor prognosis in colorectal cancer" was retracted in 2021. Reasons: duplicated images; unreliable results or conclusions; concerns about the data; concerns about the images.

## Results

### Expression of Sam68 in colorectal cancer cell lines

We examined the expression of Sam68 using Western blotting in seven human colon cancer cell lines and two cases of normal intestine tissues. The results displayed that Sam68 protein expression level was much higher in CRC cell lines than that in normal intestine tissues (Figure 1A). We next measured the expression of Sam68 mRNA in the CRC cell lines using RT-PCR (Figure 1B) and (Figure 1C). In agreement with the protein expression levels, the Sam68 mRNA expression level was much higher in CRC cell lines than that in normal intestine tissues.

**Figure 1:** **Analysis of Sam68 protein and mRNA expression in colorectal cancer (CRC) cell lines and normal intestine tissues. (A)** Analysis of Sam68 protein expression in CRC cell lines (LS174t, Colo205, SW480, HT29, HCT116, SW620) and two cases of normal intestine tissues (N1 and N2) by Western blotting. **(B)** Analysis of *Sam68* mRNA expression by RT-PCR. **(C)** Analysis of *Sam68* mRNA expression in CRC cell lines and normal intestine tissues by Q-PCR, the average ratio of *Sam68* expression normalized to *GAPDH* is shown; values are the mean ± SD of three parallel experiments.

### Sam68 is upregulated in primary human CRC lesions

Western blotting and RT-PCR analyses were performed to determine the expression of Sam68 in nine paired primary CRC tissues and the matched adjacent non-cancerous tissues. Sam68 was significantly upregulated at both the protein (Figure 2A) and mRNA levels (Figure 2B) in all nine of the CRC tissues tested, compared to the matched adjacent normal tissues from the same patient. Q-PCR results confirmed that Sam68 mRNA was upregulated in the tumor samples by up to 18.3-fold (Sam68 tumor/normal [T/N] ratio; Figure 2C; *P* < 0.01, Student’s *t*-test).

**Figure 2:** **Sam68 is upregulated in primary colorectal cancer (CRC) tissues compared with the adjacent normal tissues. (A**, **B)** Analysis of *Sam68* mRNA expression in primary CRC tissues (T) and the paired adjacent normal tissues (N) by RT-PCR **(A)** and Q-PCR **(B)**. *GAPDH* was used as loading control. **(C**, **D)** Analysis of Sam68 protein expression in primary CRC tissues and the paired adjacent normal tissues by Western blotting **(C)** and immunohistochemistry **(D)**.

In agreement with the Western blotting results, immunohistochemical analysis confirmed that Sam68 was overexpressed in all nine of the CRC tissues tested, compared with the paired adjacent normal tissues (Figure 2D). Taken together, these results indicated that Sam68 is upregulated in CRC lesions at both transcriptional and translational levels.

The article "High expression level and nuclear localization of Sam68 are associated with progression and poor prognosis in colorectal cancer" was retracted in 2021. Reasons: duplicated images; unreliable results or conclusions; concerns about the data; concerns about the images.

We further performed immunohistochemical analysis to determine the expression patterns of Sam68 in 224 paraffin-embedded CRC tissues and 43 lymph node metastatic tissues. Negative to moderate Sam68 staining was detected in the adjacent normal tissues (Figure 3A-D); however, positive Sam68 staining was detected in 206 of the 224 (92%) tumor tissues. The tumors could be divided into a low Sam68 expressing group (104 cases) and a high Sam68 expressing group (120 cases, Additional file 1: Table S1). Additionally, two main patterns of Sam68 protein expression were observed in the tumors: cytoplasmic localization (Figure 3E-F) and nuclear localization (Figure 3G-J). As shown in Additional file 1: Table S1, 61.6% (138/224) of the tumor samples displayed nuclear staining and 38.4% (86/224) displayed cytoplasmic staining. Moreover, positive expression of Sam68 was detected in 81.4% (35/43) of the lymph node metastases (Figure 4) and 65.1% (28/43) of lymph node metastases were classified as high Sam68 expressing.

**Figure 3:** **Representative images of Sam68 immunohistochemical analysis in colorectal cancer (CRC) tissues. (A** – **D)** Negative **(A**, 100X; **B**, 400X**)** or moderate **(C**, 100X; **D**, 400X**)** Sam68 staining was detected in the adjacent non-cancerous tissues. **(E** – **H)** Cytoplasmic Sam68 staining **(E**, 100X; **F**, 400X**)** or nuclear Sam68 staining **(G**, 100X; **H**, 400X**)** was observed in primary CRC tissues. **(I** – **J)** Sam68 was upregulated in CRC compared to the paired adjacent non-cancerous tissues **(I**, 100X; **J**, 400X**)**.

**Figure 4:** **Immunohistochemical analysis of Sam68 expression in metastatic lymph node tissues from colorectal cancer (CRC) patients.** Negative, moderate or strong Sam68 staining was observed in CRC metastatic lymph node tissues.

### Correlations between increased expression of Sam68 and clinical aggressiveness in CRC

Statistic analyses were performed to evaluate the expression patterns of Sam68 and the clinicopathological features of CRC. As shown in Table 1, the high Sam68 expression level was strongly correlated with poor tumor differentiation (*P* = 0.033), advanced T stage (*P* < 0.001), N stage (*P* = 0.023), and distant metastasis (*P* = 0.033) in this cohort of 224 cases of CRC. In addition, high expression level of Sam68 was significantly associated with the nuclear localization of Sam68 (*P* = 0.012). Moreover, Nuclear localization of Sam68 correlated significantly with tumor differentiation (*P* = 0.002) and advanced T stage (*P* = 0.021). These observations suggest that increased expression of Sam68 or nuclear localization of Sam68 was closely associated with aggressive phenotypes of CRC.

The article "High expression level and nuclear localization of Sam68 are associated with progression and poor prognosis in colorectal cancer" was retracted in 2021. Reasons: duplicated images; unreliable results or conclusions; concerns about the data; concerns about the images.

**Table 1:** Correlation between clinicopathologic features and Sam68 expression levels and localization

**Characteristics**	**Sam68 levels**		***P *values**	**Sam68 localization**		**R values**	***P *values**
	**Low**	**High**		**Nuclear**	**Cytoplasm**		
**Age**							
≤ mean(56)	50	56	0.833	66	40		0.848
> mean (56)	54	64		72	46		
**Gender**							
Male	61	66	0.583	76	51		0.535
Female	43	54		62	35		
**Histology**							
Columnar adenocarcinoma	79	102		110	71		0.733
Mucinous adenocarcinoma	14	11	0.083	19	6		
Others	11	7		9	9		
**Differentiation**							
Well and moderate	87	86	0.033	97	76		0.002
Poor and undifferentiated	17	34		41	10		
**T stage**							
1 ~ 2	27	13		18	22		0.021
3	58	64	<0.001	77	45		
4	19	43		43	19		
**N stage**							
0	68	59	0.023	72	55		0.072
1	27	48		50	25		
2	9	13		16	6		
**Distant metastasis**							
0 (no)	78	74	0.033	89	63		0.173
1 (yes)	26	46		49	23		
**Sam68 localization**							
Nuclear	55	83	0.012				
Cytoplasm	49	37					

### Sam68 is associated with poor prognosis in CRC patients

In univariate Cox regression analysis, tumor differentiation, T stage, N stage and distant metastasis were significant prognostic factors in this cohort of CRC patients (Additional file 2: Table S2; *P* < 0.001). Kaplan-Meier survival analysis demonstrated that patients with low levels of Sam68 expression had significantly longer median survival than patients with low Sam68 expression (Figure 5A, upper panel; 71 vs. 51 months; *P* = 0.024, log-rank test). The 5-year survival rate for patients with low Sam68 expression was 70% (95% confidence interval, 0.609-0.779), compared to 54% (95% confidence interval, 0.448-0.635) for patients with high Sam68 expression.

**Figure 5:** **Influence of Sam68 expression on overall survival in colorectal cancer (CRC). (A)** Kaplan–Meier curves showing that patients with high Sam68 expression had poorer overall survival than patients with low Sam68 expression; analysis of 224 primary CRC tissues (P = 0.003). **(B)** Kaplan–Meier curves showing that patients with high Sam68 expression in metastatic lymph node tissues had poorer overall survival than patients with low Sam68; analysis of 43 metastatic lymph node tissues (*P* = 0.029). **(C)** Kaplan–Meier curves showing that patients with nuclear Sam68 expression had poorer overall survival than patients with cytoplasmic Sam68 expression; analysis of 224 primary CRC tissues (*P* = 0.005).

The article "High expression level and nuclear localization of Sam68 are associated with progression and poor prognosis in colorectal cancer" was retracted in 2021. Reasons: duplicated images; unreliable results or conclusions; concerns about the data; concerns about the images.

Next, we analyzed the relationship between the expression of Sam68 in metastatic lymph nodes and survival. Kaplan-Meier analysis indicated that the expression level of Sam68 in the metastatic lymph nodes had a significant impact on survival (Figure 5B; *P* =0.029, log-rank test), as the median overall survival time of patients expressing low levels of Sam68 in the metastatic lymph nodes was significantly longer than patients expressing high levels of Sam68 in the metastatic lymph nodes (log-rank test, *P* = 0.029).

We also analyzed the prognostic value of the subcellular localization of Sam68 in CRC. Spearman’s rank correlation revealed that nuclear localization of Sam68 in CRC tumors correlated significantly with poorer survival (Spearman Rho −0.232, *P* = 0.001). Additionally, Kaplan-Meier survival analysis confirmed that the median survival time for patients with Sam68 nuclear localization was significantly shorter than patients with Sam68 cytoplasmic localization (Figure 5C; 54 vs. 73 months, *P* = 0.024, log-rank test). The 5-year survival rate for patients with Sam68 cytoplasmic localization was 70% (95% confidence interval, 0.609-0.779), compared to 54% (95% confidence interval, 0.448-0.635) for patients with Sam68 nuclear localization. The Sam68 expression level, subcellular localization of Sam68, pathological stage and N stage were identified as independent prognostic factors for overall survival in CRC in multivariate survival analysis (Additional file 3: Table S3 and Additional file 4: Table S4).

Furthermore, in the subgroups of CRC patients without distant metastasis (M0) or with well/moderately differentiated tumors, both the Sam68 expression level (Figure 6A and C) and subcellular localization of Sam68 (Figure 6E and G) correlated significantly with overall survival. However, no such correlations were observed in the subgroup of patients with distant metastasis or poorly differentiated tumors (Figure 6B,D,F and H).

**Figure 6:** **Overall survival curves for colorectal cancer (CRC) patients stratified by the Sam68 expression level, according to M classification and tumor differentiation.** In the M0 classification **(A)** and moderately differentiated tumor subgroups **(C)**, patients with low Sam68 expression had significantly better overall survival than patients with high Sam68 expression (*P* = 0.01). In the M1 classification **(B)** and poorly differentiated tumor subgroups **(D)**, the overall survival of patients with high and low Sam68 expression was not significantly different. In the M0 classification **(E)** and moderately differentiated tumor subgroups **(G)**, patients with Sam68 cytoplasmic localization had significantly better overall survival (*P* = 0.027 and *P* = 0.024, respectively) than patients with Sam68 nuclear localization. In the M1 classification **(F)** and poorly differentiated subgroups **(H)**, the overall survival of patients with Sam68 cytoplasmic and nuclear localization was not significantly different.

The article "High expression level and nuclear localization of Sam68 are associated with progression and poor prognosis in colorectal cancer" was retracted in 2021. Reasons: duplicated images; unreliable results or conclusions; concerns about the data; concerns about the images.

## Discussion

Sam68 is a substrate of the oncogenic Src kinase, which is often activated in human cancers [4]. Previous researches suggested that two opposing functions of Sam68 were reported in different cellular contexts. On one hand, a few studies indicated that Sam68 acted as a tumor suppressor. For example, Sam68 deficiency resulted in neoplastic transformation of murine NIH3T3 fibroblasts. Reduction of Sam68 was associated with anchorage-independent growth, defective contact inhibition, and the ability to form metastatic tumors in nude mice [31], while overexpression of Sam68 in NIH-3 T3 fibroblasts led to both cell cycle arrest and apoptosis [21]. On the other hand, a large proportion of recent reports demonstrated that Sam68 played an oncogenic role. Sam68 knockdown in polyoma middle T-antigen (PyMT) oncogene transformed cell lines delayed tumorigenesis and metastasis formation in nude mice [25]. Busà R and colleagues have demonstrated that Sam68 was upregulated in prostate cancer at both protein and mRNA levels. Additionally, downregulation of Sam68 in prostate cancer cells delayed cell cycle progression and reduced the proliferation rate [23]. Sam68 is also upregulated and its upregulation is correlated with shorter survival rates in breast cancer, cervical cancer, renal cell carcinoma [24,27,28]. The present study demonstrated that Sam68 was elevated in CRC tissues and the high Sam68 expression level was significantly correlated with the characteristics of aggressive CRC (including poor differentiation of tumors, advanced T stage, lymph node involvement and distant metastasis). Additionally, high Sam68 expression level was a significant predictor of poor prognosis in CRC patients. Thus, our results raised the evidence that suggested that Sam68 might promote development and progression of human CRC, supporting the pro-oncogene role of Sam68 in human cancer.

Sam68 is a ubiquitously expressed protein and resides in both cytoplasm and nuclei [2]. Posttranslational modifications of Sam68, such as phosphorylation and methylation, can affect its subcellular localization, interaction with signaling proteins, as well as affinity for target RNAs [2,15,32-35]. In most cells, Sam68 predominantly resided within the nucleus and is involved in gene transcription, alternative splicing, and nuclear export [12-19]. Sam68 has been observed to exist in dynamic nuclear foci termed Sam68 nuclear bodies (SNBs), also called stress nuclear bodies [12,36]. Genes regulated by Sam68 include CD44, Bcl-xl, Sgce, SMN2, SF2/ASF, Cyclin D1, and so on, which are all involved in oncogenesis [6,14-19]. In the present study, Sam68 was found to localize to both the nuclei and cytoplasm of cancer cells. It is particularly noteworthy that the subgroup of patients with advanced clinical stage CRC often exhibited nuclear localization of Sam68, while CRC patients with well differentiated or early stage tumors often displayed cytoplasmic Sam68 staining. In addition, patients with cytoplasmic Sam68 localization had a better clinical outcome than patients with Sam68 nuclear localization. These researches suggested that nuclear Sam68 might play a dominant role in oncogenesis of CRC. However, distinguished from our results, cytoplasmic localization of Sam68 was significantly correlated with cancer progression and poor prognosis in human renal cell carcinoma and breast cancer [24,27]. It could be due to the functions of Sam68 in multiple signaling pathways, since it can be expressed in both the cytoplasm and nucleus. In the cytoplasm, Sam68 interacts with signaling molecules such as Src, Grb2, Grap [7-11] and stimulates oncogenic pathways, including the epidermal growth factor pathway, ERK and AKT pathways [37,38]. In renal cell carcinoma and breast cancer, the oncogenic role of Sam68 was closely associated with its activation of Akt/GSK-3β pathway [24,27]. Taken together, these researches suggested that cytoplasmic and nuclear localization of Sam68 might contribute to neoplastic transformation or tumor progression through different molecular mechanisms in different cancer types or cellular contexts.

The article "High expression level and nuclear localization of Sam68 are associated with progression and poor prognosis in colorectal cancer" was retracted in 2021. Reasons: duplicated images; unreliable results or conclusions; concerns about the data; concerns about the images.

This study provides the first evidence to indicate that both high expression level and nuclear localization of Sam68 correlate significantly with invasiveness and aggressiveness characteristics in CRC, and poorer survival of CRC patients. Taken together, this study suggests that Sam68 may represent a novel indicator of progression and prognosis in CRC.

## Conclusions

In conclusion, Sam68 was upregulated in primary human CRC, and high Sam68 expression levels in CRC were associated with the clinical features of aggressive disease and poorer patient prognosis. Nuclear localization of Sam68 in CRC was identified as an independent predictor of poor prognosis. However, further characterization of the mechanisms by which Sam68 is involved in the transformation and progression of human CRC is required.

## Competing interests

The authors declare that they have no competing interests.

## Authors’ contributions

WTL participated in the design of the study and drafted the manuscript. JLL and ZGW carried out the experiment of cell culture and molecular biology. LS supported the statistical analysis. YMC and TTL supported the evaluation of the immunohistochemical results. XHZ and XTC participated in collecting the clinical samples. LBS and YQD participated in the design of the study. All authors read and approved the final manuscript.

The article "High expression level and nuclear localization of Sam68 are associated with progression and poor prognosis in colorectal cancer" was retracted in 2021. Reasons: duplicated images; unreliable results or conclusions; concerns about the data; concerns about the images.

## Pre-publication history

The pre-publication history for this paper can be accessed here:

http://www.biomedcentral.com/1471-230X/13/126/prepub

## Supplementary Material

Additional file 1: Table S1 Clinicopathologic variables for patient cohort (n = 224). Click here for file

Additional file 2: Table S2 Univariate Cox regression analysis of potential prognostic factors for CRC patients. Click here for file

Additional file 3: Table S3 Multivariate Cox regression analysis of Sam68 levels and other potential prognostic factors for CRC patients. Click here for file

Additional file 4: Table S4 Multivariate Cox regression analysis of Sam68 localization and other potential prognostic factors for CRC patients. Click here for file
